RETRACTED

# Biomolecule Protective and Photocatalytic Potential of Cellulose Supported MoS_2_/GO Nanocomposite

**DOI:** 10.1155/2023/3634726

**Published:** 2023-03-09

**Authors:** Muhammad Pervaiz, Muti Ur Rehman, Faisal Ali, Umer Younas, Mika Sillanpaa, Rizwan Kausar, Asma A. Alothman, Mohamed Ouladsmane, Mohammad Abdul Mazid

**Affiliations:** ^1^Department of Chemistry, Government College University, Lahore, Pakistan; ^2^Department of Chemistry, The University of Lahore, Lahore, Pakistan; ^3^Department of Biological and Chemical Engineering, Aarhus University, Nørrebrogade 44, Aarhus 8000, Denmark; ^4^Department of Chemistry, Kallar Kahar Science College, Kallar Kahar, Chakwal, Pakistan; ^5^Department of Chemistry, College of Science, King Saud University, Riyadh 11451, Saudi Arabia; ^6^Department of Pharmaceutical Chemistry, Faculty of Pharmacy, University of Dhaka, Dhaka 1000, Bangladesh

## Abstract

In the current study, cellulose/MoS_2_/GO nanocomposite has been synthesized by a hydrothermal method. Reports published regarding efficiency of Mo and graphene oxide-based nanocomposites for environmental remediation motivated to synthesize cellulose supported MoS_2_/GO nanocomposite. Formation of nanocomposite was initially confirmed by UV-visible and FTIR spectroscopic techniques. Particle size and morphology of the nanocomposite were assessed by scanning electron microscopy (SEM), and it was found having particle size ranging from 50 to 80 nm and heterogeneous structure. The XRD analysis also confirmed the structure of the nanocomposite having cellulose, MoS_2_, and GO. The synthesized nanocomposite was further tested for biomolecule protective potential employing different radical scavenging assays. Results of radical DPPH^●^ (50%) and ABTS^**●+**^ (51%) scavenging studies indicate that nanocomposites can be used as a biomolecule protective agent. In addition, nanocomposite was also evaluated for photocatalytic potential, and the results showed excellent photocatalytic properties for the degradation of 4-nitrophenol up to 75% and methylene blue and methyl orange up to 85% and 70%, respectively. So, this study confirmed that cellulose supported/stabilized MoS_2_/GO nanocomposite can be synthesized by an ecofriendly, cost-effective, and easy hydrothermal method having promising biomolecule protective and photocatalytic potential.

## 1. Introduction

Environmental pollution is increasing day by day due to different industrial activities and urbanization, and hydrosphere has become badly polluted [1]. These pollutants are harmful for human beings and aquatic life as well [2]. According to an estimate, 50% of the world's population has been facing the scarcity of water and 900 million people have been deprived of the fresh water resources. Due to the polluted water, about 6 million people and 1.8 million children die every year due to different waterborne diseases. Pakistan is facing the same issue of water pollution due to poor sanitation system, industrialization, and urbanization [3]. The most common sources of water pollution are industries such as textile, paper and pulp, and leather. A huge amount of industrial effluent is being discharged by industries to water streams. [4]. Industrial effluent usually contains toxic chemicals especially dyes that can cause a lot of damage to humans and aquatic animals. There are so many techniques and methodologies which are being applied in different countries of the world for the removal of dyes from the aqueous medium [5], and nanotechnology is one of the best among all of those. Therefore, nanomaterials including metal nanoparticles and graphene oxide-based nanocomposites having small size and large surface area can be used for wastewater treatment [6, 7]. Metal nanoparticles Fe, Ag, metal oxides (TiO_2_, V_2_O_5_) nanoparticles, and nanocomposites have been synthesized for the catalytic removal of dyes from wastewater [8, 9].

RETRACTED

Research studies have reported the antioxidant role of molybdenum nanoparticles along with photocatalytic applications for the degradation of ketamine [10]. Presence of free radicals and reactive oxygen/nitrogen species can damage biomolecules in the human body and instigate many diseases. Deterioration in lipid-containing food products or any other biomaterial may appear due to presence of free radicals or reactive species [11]. Free radical scavenging compounds are very helpful as they stop the oxidation process and protect biomolecules from damage. Nowadays, scientists have been using multiple compounds (synthetic, natural, and nanoparticles) as antioxidants to overcome this problem [12, 13].

These days, the synthesis of nanoparticles by green/simple, cost-effective methods has gained attention, and now, there is a big need to use the fast and cost-effective methods for the synthesis of nanomaterials [14, 15]. Keeping in view the importance of nanocomposites as catalytic and radical scavenging materials, cellulose-supported MoS_2_@GO nanocomposite has been synthesized. Synthesis was planned to be performed using a simple and fast hydrothermal method by avoiding excessive use of chemicals. Characterization was conducted by UV-visible, FTIR, SEM, and XRD techniques. The nanocomposite was then tested for the degradation of 4-nitrophenol which is an organic pollutant that is usually discharged by pharmaceutical industries and two dyes that are found in textile industry effluents. In addition, photocatalytic potential of the nanocomposite was determined for the degradation of selected dyes. Biomolecule protective efficiency was tested by measuring radical scavenging potential of nanocomposite employing DPPH^●^ and ABTS^**●+**^ assays. This research work will motivate the researchers working on synthesis and applications of nanomaterials to prefer the methods that need relatively less efforts, use of chemicals, and resources.

RETRACTED

## 2. Materials and Methods

### 2.1. Chemicals and Reagents

Methylene blue (99.99%) was purchased for the Fisher Scientific UK; methyl orange (99.9%) was purchased from the Sigma Aldrich from Germany. Cellulose, graphite, ammonium molybdenite, hydrogen peroxide, sodium nitrate, hydrochloric acid, ethanol, 4-nitrophenol, and nitric acid were also purchased from the Sigma Aldrich from Germany. All the reagents were of analytical grade, and no further purification was needed for laboratory use.

### 2.2. Synthesis of Cellulose Nanofiber

Cellulose nanofiber was prepared by socking soft wood pulp sheet in water on a hot plate for 12 hours at 25°C (Figure 1(a)). Then, swollen pulp was disintegrated for 10–20 min using a blender. The resulting slurry was then added to a conical flask, Zirconia balls were added, and milling was conducted at 100°C for 4 h. Nanofibers of cellulose were obtained and used for the synthesis of nanocomposite [16].

### 2.3. Synthesis of MoS_2_ Nanoparticles (Centrifuging Method)

Nanoparticles (NPs) of MoS_2_ were prepared (Figure 1(b)) using ammonium molybdenite as a precursor. In 50 mL of acetic acid, 1.3 g of ammonium molybdenite was added followed by adding 100 mL of distilled water. It was placed on a hot plate with continuous stirring at 90°C for 30 min, and then ammonia water was added to it and stirred for further 4 h at 50°C. In the resulting mixture, 2 g of urea was added and stirring was done for 5 min to form the gel type material. Viscous solution (40 mL) was transferred into the autoclave, and temperature was kept at 160°C for 10 h. After removing the autoclaved solution from the oven, it was cooled for 5 h at room temperature. Centrifugation was performed at 40 rpm for 30 min, and precipitates were collected and washed with distilled water and ethanol to remove impurities. The final product was obtained after drying in the oven [16].

### 2.4. Synthesis of GO Nanoparticles (Modified Hammer Method)

Graphene oxide was synthesized employing the modified Hammer's method (Figure 1(c)). Graphite (5 g) and NaNO_3_ (2.5 g) were mixed in a beaker (mixture A). In another beaker, 105 mL of sulphuric acid and 12 mL of H_3_PO_4_ were mixed (mixture B). Mixture A was poured into mixture B and after mixing placed on an ice bath for 10 min. In the resulting mixture, 15 g of KMnO_4_ was added and temperature was maintained below 5°C for 60 min. As a result, suspension was obtained. The solution was then removed from ice bath and placed on stirrer 98°C with continuous addition of water. After sometime, 15 mL of H_2_O_2_ was added to the reaction mixture and centrifuged at 4000 rpm for 30 min. The final product was washed with distilled water and 20% HCl for three times to get the GO nanoparticles [17, 18].

RETRACTED

### 2.5. Synthesis of Cellulose/MoS_2_/GO Nanocomposite (Hydrothermal Method)

Nanocomposite cellulose/MoS_2_/GO was synthesized (Figure 1(d)) by a two-step process. In the first step, 2 grams of cellulose nanoparticles and 1 gram of MoS_2_ in distilled water were used followed by stirring for 60 min in a hot plate. A viscous solution of cellulose and MoS_2_ appeared. It was shifted to the autoclave and heated in the oven at 200°C for 4 h. After 4 h, the autoclave was cooled to room temperature. Centrifugation was performed, and precipitates were separated at 35000 rpm for 20 min. Precipitates were washed with distilled water/ethanol for three times and dried at room temperature for three days. In the second step, cellulose/MoS_2_ was dissolved in distilled water and 0.5 g of GO was mixed. The resulting mixture was heated 50°C for 2 h followed by sonication for 10 min. After sonication, 100 mL of material was shifted to the autoclave and transferred to the oven at 300°C for 4 h. The autoclave was then cooled at 25°C for 4 h, and centrifugation was conducted for 30 min. The precipitates were collected and washed with distilled water and ethanol for three times to remove all types of impurities. The final product was dried for 7 days at room temperature to get the grey color cellulose/MoS_2_/GO nanocomposite.

### 2.6. Characterization

The characterization of the synthesized nanoparticles and nanocomposite was conducted with the help of UV-visible (CECIL 7400-ce Aquarius Cambridge, UK) and FTIR spectrophotometer (Bruker alpha (II), UK). The scanning electron microscopic (SEM) analysis was performed using NOVA FE- SEM 450. The X-ray diffraction (XRD) analysis of the nanocomposite was also performed using the Bruker diffractometer (Coventry, UK). Characterization confirmed the formation of nanoparticle and nanocomposite.

### 2.7. Biomolecule Protective Potential

Biomolecule protective potential of the nanocomposite was evaluated in terms of free radical (DPPH^●^ and ABTS^●**+**^) scavenging activities. Antioxidant activities of nanocomposite cellulose/MoS_2_@GO were determined using DPPH^●^ and ABTS^●**+**^ assays. One milligram of nanocatalyst was added separately to the test tube solution containing 1 mL of DPPH^●^ (0.01 mM) and ABTS^●+^ (0.03 mM) followed by addition of 5 mL of methanol and 4 mL of water. The scavenging of free radicals was determined by recording their spectra using a UV-visible spectrophotometer after regular intervals. Percentage scavenging formula = (*A*_*d*_ − *A*_*s*_/*A*_*d*_) × 100. Here, *A*_*d*_ is the absorbance of pure DPPH^●^ and ABTS^●**+**^ solutions, and *A*_*s*_ is the absorbance of the sample [13, 19].

RETRACTED

### 2.8. Photocatalytic Potential of Cellulose/MoS_2_/GO

Photocatalytic potential of the nanocomposite was determined in terms of its dye degradation potential under sunlight by following a method reported earlier [20]. Solutions of dyes such as methylene blue (1 mM) (*λ*_max_ value of 667 nm) and methyl orange (1 mM) (*λ*_max_ of 467 nm) were prepared. Catalytic degradation of methylene blue was carried out in direct sunlight by taking 0.01 mM solution of methylene blue in 5 different test tubes having 1, 3, 5, 7, and 10 milligram of catalyst being added to them, and the tubes were placed in direct sunlight. Degradation was observed using a UV-visible spectrophotometer after regular intervals. In the same way, catalytic degradation of methyl orange was also performed and results were recorded [21]. Another organic pollutant, i.e., 4-nitrophenol, commonly found in pharmaceutical effluent, was degraded using cellulose/MoS_2_/GO. Solution of 4-nitrophenol solution was prepared by adding its 0.0139 gram in 100 mL of water to get 1 mM solution having *λ*_max_ at 400 nm. The degradation of 4-nitrophenol was also performed under sunlight in 5 different test tubes with 5 mL 1 mM solution, and degradation was recorded using a UV-visible spectrophotometer [22].

## 3. Results and Discussion

### 3.1. UV-Visible Analysis

Analysis of all the products including cellulose nanofiber, GO, MoS_2_, and cellulose/MoS_2_/GO nanocomposite was performed by using a UV-visible spectrophotometer. In UV-visible analysis, the observed value for cellulose appeared at 358 nm, comparable with the already reported value at 360 nm [23] (Figure 2(a) (i)). The UV-visible spectra for MoS_2_ was also recorded, and a peak was observed at 345 nm which was close to the reported value 340 nm [24] that confirmed the formation of MoS_2_ nanoparticles (Figure 2(a) (ii)). In UV-visible analysis, GO showed a peak at 355 nm which is in close resemblance with an already reported value at 350 nm as shown in Figure 2(a) (iii). Nanocomposite, i.e., cellulose/MoS_2_/GO, was also analyzed using a UV-visible spectrophotometer, and spectra were obtained having a peak at 348 nm which does not resemble with any spectra of the individual component (cellulose, MoS_2_, and GO). It confirms the association of all the components involved in nanocomposites, as it lies in between the values of nanoparticles and the nanocomposite (Figure 2(a) (iv)).

RETRACTED

The plot between (ahv)^1/2^ vs. energy (eV) presenting the band gap of nanocomposites, MoS_2_ NPs and GO. The GO has the highest energy band gap (3.90 eV), while MoS2/GO have intermediate and it was found having the lowest energy band gap. It reveals that nanocomposite can easily provide electrons necessary to be available for photocatalysis, and the same results have been reported in previous studies [25]. Correspondingly, nanocomposites with GO showed a similar band gap energy of 3.52 eV as reported earlier [26].

### 3.2. Fourier Transform Infrared Analysis

The FTIR analysis of cellulose nanofiber, GO, MoS_2_, and cellulose/MoS_2_/GO nanocomposite was performed. In Figures 3 (a)–(d), spectra for cellulose nanofiber, MoS_2_, GO nanoparticles, and cellulose/MoS_2_/GO nanocomposite have been presented. FTIR spectra revealed different identities of nanoparticles as well as nanocomposite. In Figure 3 (a), (cellulose nanofiber) peak at 800 cm^−1^ shows the presence of an aromatic compound [27], a broad absorption band at 3,333–3,400 cm^−1^, which corresponds to hydroxyl group (–O–H stretching) vibrations in cellulose [28]. Another peak observed at 1,057 cm^−1^ may be due to skeletal vibration in –C–O–C and *β*-glycosidic at 897 cm^−1^ [29]. Formation of MoS_2_ nanoparticles was confirmed by the FTIR analysis (Figure 3 (b)) that shows different peaks as representative of MoS_2_ nanoparticles. A stretching peak observed around 610 cm^−1^ can be attributed to the stretching of Mo-S bond [30, 31]. The spectrum recorded for GO (Figure 3 (c)) was found containing broad band around 3,400 cm^−1^ that is a strong indication of OH stretching. Second, a peak around 1,600 cm^−1^ indicates the stretching of C=C, and peaks at 1,800 cm^−1^, 1,200 cm^−1^, and 1,020 cm^−1^ may be due to the presence of C=O, C-OH, and C-O, respectively [32, 33].

In Figure 3 (d), the FTIR spectrum recorded for nanocomposite (cellulose/MoS_2_/GO) has been presented. All the characteristic peaks of cellulose nanofiber, MoS_2_ nanoparticles, and GO were obtained in the spectrum of the nanocomposite. It confirms the association among all the components of the nanocomposite. The peak for skeletal vibration in –C–O–C was observed at 1,057 cm^−1^, and a band appearing at 590 cm^−1^ indicated the presence of Mo-S and S-S linkage. In addition, representative peaks of GO can also be observed in the spectrum. All the evidence obtained after FTIR spectra confirmed the formation of not only precursors but the nanocomposite as well.

RETRACTED

### 3.3. XRD Studies

XRD analysis shows (Figure 4) the formation of nanocomposite cellulose/MoS_2_/GO. The graph is shown between 2*θ* along *x*-axis and intensity along *y*-axis by comparison of different Miller index values. It is concluded on the basis of the graph that crystalline structure exhibited Miller indexes values as 002, 110, 004, 101, 102, 103, 006, 105, 105, 105, 110, 112, 107, 114, 202, 203, and 116 at 2*θ* 14.39°, 29.014°, 32.80°, 33.62°, 35.98°, 39.65°, 44.14°, 49.87°, 56.07°, 58.55°, 60.64°, 62.85°, 66.66°, 68.76°, 69.24°, 70.68°, 73.04°, 76.31°, 77.54°, 78.15°, and 80.44°, respectively (Table 1). The curve at 22.45° shows the amorphous presence of cellulose, and at 26.34°, (110) represents GO with orthorhombic crystalline nature. XRD studies confirmed the formation of nanocomposite [34]. The nanocomposite crystalline phase was hexagonal with PDF#73-1508. The crystallite size was 6.447 nm using Debye Scherrer equation *D* (nm) = *kλ*/*β* cos*θ*, where *D* (nm) represents crystallite size, *k* denotes constant, *β* is full-width half maximum, and *θ* is the angle. The details of hkl and interplanar distance (Å) with 2*θ* are mentioned in Table 1. Likewise, results were also reported by some researchers recently [35, 36].

### 3.4. SEM Analysis

The size and morphology of nanocomposite was evaluated by scanning electron microscopy. The SEM images (Figure 5) were taken at different resolutions. The diameter of synthesized nanocomposite was noted up to 50–80 nanometres having a heterogeneous surface. Such surface of the synthesized nanocomposite may be suitable if it is used as a photocatalyst for degradation of dyes [37]. The nanoparticles of MoS_2_ stabilized by cellulose can be clearly seen at the surface of GO (Figure 5(a)), and the GO nanosheet's surface without cellulose stabilized nanoparticle loading is shown in Figure 5(b). GO nanosheet's surfaces have high porosity which are available for the fitment of cellulose stabilized MoS_2_ NPs.

### 3.5. Photocatalytic Potential of Cellulose/MoS_2_/GO

Photocatalytic potential of the nanocomposite was evaluated in terms of degradation of the selected toxic pollutants. The nanocomposite was used as a catalyst to carry out the degradation process in a smooth and accelerated manner. A pollutant 4-nitrophenol was subjected to degradation using cellulose/MoS_2_/GO nanocomposite under sunlight, and results have been shown in the Figure 6. Results show that the catalyst has significantly contributed towards degradation of 4-nitrophenol. In the absence of the catalyst, degradation was not observed, and after adding the nanocomposite, degradation of 4-nitrophenol up to 75% was achieved just in 12 min. Graphene oxide in combination with MoS_2_ has been reported for the degradation of 4-nitrophenol [38, 39].

RETRACTED

Many researchers have reported the use of MoS_2_-based nanomaterials for the degradation of dyes from different effluents [40]. In the same way, degradation of methylene blue was achieved using the nanocomposite under sunlight directly. Photocatalytic degradation was observed at *λ*_max_ 667 nm using a UV-visible spectrophotometer. The degradation was started after adding the nanocomposite, and maximum degradation up to 85% was achieved in 10 min (Figure 7). Results of the current study may be considered better in comparison with already reported for the degradation of methylene blue dye using molybdenum-based nanomaterials [41].

The role of molybdenum-based nanomaterials for the removal of organic contaminants has already been reported in many studies [42]. The degradation of methyl orange was also performed under sunlight directly, and the process was observed using a UV-visible spectrophotometer at *λ*_max_ of 467 nm. Degradation of the dye takes place after adding the nanocomposite to the dye solution. Degradation up to 70% was achieved (Figure 8) that is comparable with the degradation potential of molybdenum composite, already reported for methyl orange [43].

### 3.6. Biomolecule Protective Potential

Reports revealed that MoS_2_ nanomaterials can be used for the removal of reactive oxygen species that are responsible for oxidative stress and biomolecule damages [44]. Biomolecule protective potential of the nanocomposite has been determined by evaluating radical (DPPH^●^ and ABTS^●**+**^) scavenging potential. The DPPH^●^ assay was performed, and the nanocomposite was allowed to react with DPPH free radicals. Decrease in concentration of free radicals was observed using a UV-visible spectrophotometer at 530 nm after regular interval of times (Figure 9). Decrease in absorbance of the solution indicated the scavenging of free radicals, and the maximum amount of radicals (45%) was neutralized by the nanocomposite in 24 min. The remaining amount of the free radicals can be removed using a high concentration of the nanocomposite. MoS_2_-based nanocomposite synthesized in the current study exhibited improved DPPH radical scavenging potential as compared to that reported earlier [45].

With the help of cellulose/MOS_2 /_GO, the radical scavenging of ABTS^●**+**^ was determined. Radical scavenging was observed with the help of a UV-visible spectrophotometer at 651 nm. The nanocomposite exhibited maximum radical scavenging potential in 49 min, and 45% of the radicals were neutralized (Figure 10).

RETRACTED

Comparative potential of the nanocomposite for the removal of selected dyes and free radicals has been presented in Table 1. It is clear that nanocomposite is potent enough for the catalytic degradation methylene blue as compared to other two dyes. However, the efficiency of the nanocomposite for the neutralizing free radicals was found to be same. The efficiency of cellulose/MoS_2_/GO for the removal of dyes/free radicals has been compared with the other molybdenum-based nanoparticles/nanocomposite. Removal efficiency was found to be lesser as compared to the previously reported data. It may be due to the cellulosic material Table 2 covering around MoS_2_ and GO.

## 4. Conclusion

Synthesis of nanomaterials has been focused by many researchers due to their vast spectrum of applications. Most of the scientists are focusing to synthesize nanomaterials by simple methods with lesser involvement of toxic chemicals. This target has been achieved by synthesizing cellulose/MoS_2_/GO nanocomposite material by the simple, ecofriendly, and cost-effective hydrothermal method without compromising on activity potential. This work will provide a path for the researchers to adopt simple methodologies for the fabrication of nanomaterials of their interest. The synthesized nanocomposite was found having size ranging from 50 to 80 nm and heterogeneous structure. It was found active against ABTS^●+^ and DPPH^●^, providing an evidence for its biomolecule protective nature. In addition, degradation of 4-nitrophenol, methylene blue, and methyl orange was catalyzed by cellulose/MoS_2_/GO, and the results confirmed photocatalytic potential of the nanocomposite. Authors strongly recommend the hydrothermal synthesis method for the fabrication of nanomaterials. Nanocomposite cellulose/MoS2/GO synthesized in this study can be used for the protection of biomolecules from free radicals. It can also be used as a nanocatalyst for the removal of 4-nitrophenol found in pharmaceutical effluent and dyes from textile industry wastewater.

## Figures and Tables

**Figure 1:** (a) Synthesis of cellulose NPs. (b) Synthesis of MoS_2_ NPs. (c) Synthesis of GO nanoparticles. (d) Synthesis of cellulose/MoS_2_/GO NCs.

**Figure 2:** (a) UV-visible spectra: (i) cellulose nanofiber, (ii) MoS_2_ nanoparticles, (iii) GO, and (iv) cellulose/MoS_2_/GO nanocomposite; (b) band gap energy.

**Figure 3:** FTIR spectra: (a) cellulose nanofiber, (b) MoS_2_ nanoparticles, (c) GO, and (d) cellulose/MoS_2_/GO nanocomposite.

**Figure 4:** XRD studies of cellulose/MoS_2_/GO.

**Figure 5:** SEM images of cellulose/MoS_2_/GO nanocomposite.

RETRACTED

**Figure 6:** Photocatalytic degradation of 4-nitrophenol using cellulose/MoS_2_/GO, %age degradation (inset).

**Figure 7:** Photocatalytic degradation of methylene blue using cellulose/MoS_2_/GO, %age degradation (inset).

**Figure 8:** Photocatalytic degradation of methyl orange using cellulose/MoS_2_/GO, %age degradation (inset).

**Figure 9:** DPPH radical scavenging potential of cellulose/MoS_2_/GO, % inhibition (inset).

**Figure 10:** ABTS radical cation scavenging potential of cellulose/MoS_2_/GO, % inhibition (inset).

**Table 1:** XRD data of cellulose/MoS_2_/GO nanocomposite.

2 theta	*d* (Å)	hkl	FWHM
14.39	6.15	(0 0 2)	0.46
29.014	3.075	(0 0 4)	0.077
32.803	2.728	(1 0 0)	0.244
33.623	2.6633	(1 0 1)	0.101
35.985	2.4937	(1 0 2)	0.277
39.651	2.2712	(1 0 3)	0.247
44.141	2.05	(0 0 6)	0.19
49.875	1.8269	(1 0 5)	0.298
56.071	1.6388	(1 0 6)	0.343
58.559	1.575	(1 1 0)	0.394
60.132	1.5375	(0 0 8)	0.4
60.643	1.5258	(1 1 2)	0.231
62.858	1.4772	(1 0 7)	0.37
66.663	1.4018	(1 1 4)	0.422
68.766	1.364	(2 0 0)	0.089
69.248	1.3557	(2 0 1)	0.107
70.211	1.3394	(1 0 8)	0.16
70.683	1.3316	(2 0 2)	0.299
73.047	1.2943	(2 0 3)	0.451
76.157	1.249	(1 1 6)	0.153
76.31	1.2468	(2 0 4)	0.123
77.547	1.23	(0 0 10)	0.248
78.159	1.2219	(1 0 9)	0.288
80.44	1.1929	(2 0 5)	0.319

**Table 2:** Comparative potential of cellulose/MoS_2_/GO for the removal of dyes/free radicals.

Present work					Previous literature	
Sr. no.	Dye/free radical removal	Process/mechanism	Removal efficiency (%)	Time (min)	Nanocomposite	Removal efficiency
1	4-nitrophenol	Photocatalytic degradation	75	12	Molybdenum doped titania semiconductors	90% [46]
2	Methylene blue	Photocatalytic degradation	85	10	Titanium dioxide-molybdenum disulfide	90% [47]
3	Methyl orange	Photocatalytic degradation	70	120	Molybdenum-modified titanium dioxide	84% [48]
4	DPPH^●^	Electron transfer	45	24	Molybdenum oxide-Starbon	50% [49]
5	ABTS^●**+**^	Electron transfer	45	49	Molybdenum trioxide nanoparticles	80% [12]

## Data Availability

No data were used to support the findings of this study.
